# Modelling the Latent Semantics of Diffusion Sources in Information Cascade Prediction

**DOI:** 10.1155/2021/7880215

**Published:** 2021-09-29

**Authors:** Ningbo Huang, Gang Zhou, Mengli Zhang, Meng Zhang, Ze Yu

**Affiliations:** State Key Laboratory of Mathematical Engineering and Advanced Computing, Zhengzhou 450001, China

## Abstract

Predicting the information spread tendency can help products recommendation and public opinion management. The existing information cascade prediction models are devoted to extract the chronological features from diffusion sequences but treat the diffusion sources as ordinary users. Diffusion source, the first user in the information cascade, can indicate the latent topic and diffusion pattern of an information item to mine user potential common interests, which facilitates information cascade prediction. In this paper, for modelling the abundant implicit semantics of diffusion sources in information cascade prediction, we propose a Diffusion Source latent Semantics-Fused cascade prediction framework, named DSSF. Specifically, we firstly apply diffusion sources embedding to model the special role of the source users. To learn the latent interaction between users and diffusion sources, we proposed a co-attention-based fusion gate which fuses the diffusion sources' latent semantics with user embedding. To address the challenge that the distribution of diffusion sources is long-tailed, we develop an adversarial training framework to transfer the semantics knowledge from head to tail sources. Finally, we conduct experiments on real-world datasets, and the results show that modelling the diffusion sources can significantly improve the prediction performance. Besides, this improvement is limited for the cascades from tail sources, and the adversarial framework can help.

## 1. Introduction

With the fast development of information technology and mobile communication technique, online media such as social networks and news platforms have become an indispensable way for people to acquire information and deeply influence the economy and culture. Information diffusion is a common phenomenon in the real world, such as the retweet of tweets in social network, the paper citation in academic network, and the spread of epidemic. The information diffusion on the online media is faster, deeper, wider, and harder to control compared with traditional media such as newspapers and broadcasts [1]. Hence, for public opinion government [2, 3] and marketing [4–8], it is important to mine the law behind information diffusion on online media [5]. In the past decade, researchers begin to predict the future trends in information diffusion [9–19]. The prediction can be divided into two aspects such as user-level prediction and cascade-level prediction according to the granularity of predicted targets. Cascade-level prediction focuses on the global characteristics of the whole cascade such as the increment size [14, 17] and the popularity [9, 10, 18, 19]. User-level prediction focuses on the microuser behaviour in the network who will be the next user retweet this post.

Our work focuses on user-level prediction, that is, the next active user prediction. In earlier years, researchers manually extract features including sequences, social context, and information items features from information cascade [10]. However, feature-based models require abundant expert knowledge and complicated feature extraction. Recently, with the fast development of deep learning techniques, diffusion prediction methods based on deep sequence models have emerged. Recurrent neural network (RNN) is a classical deep learning model for sequence modelling. Its variants such as gated recurrent unit (GRU) [20] and long short-term memory (LSTM) [21] are widely used in applications such as natural language process [22] and anomaly detection [23]. In information cascade prediction, RNN-based models encode the sequence into a low dimension vector and predict the next user based on the sequence encoding. However, the RNN-based models suffer from the long-term dependency problem. To address this problem, DeepDiffuse [12] introduces attention mechanism [22] to focus on the subsequences which contribute most to cascade prediction. Another problem of RNN-based models is that RNN must be calculated sequentially and is hard to be parallelized. The self-attention model [24] alleviates this problem, and DAN [25] and HiDAN [26] adopt the hierarchical attention model to capture the cross-dependency efficiently and effectively. Besides, some research studies also take the social relationship into consideration by using the LSTM variants [13, 27, 28] or graph neural network [29, 30].

Previous methods [12, 13, 25–28] only extract the chronological feature of the cascade sequences but ignore the heterogeneity of different information. It is unreasonable in the real world because users show different interests in different information items. And, users' diffusion behaviours could be diverse according to the types of information. Though some methods [31] based on the independent cascade (IC) can model the information heterogeneity with topic modelling, sometimes the information contents are hard to collect [32]. Fortunately, we can mine abundant semantics behind the diffusion sources to model the heterogeneity of information items, which can facilitate information cascade prediction. On the one hand, diffusion sources can indicate the potential activated user group of information: in social network, as shown in Figure 1(b), in the broadcast diffusion of social network, users are more likely to directly forward the tweets from diffusion sources [33]. This kind of diffusion usually comes from very influential diffusion sources who have large numbers of followers [34], and the potential activated user group should be closely related to the source user. However, in word-to-mouth diffusion, users tend to retweet from their friends, and in this case, the potential activated user group will be closed to the last activated user. In academic network, researchers tend to directly follow the influential scholars, while the less well-known research studies are usually spread by others' citation. On the other hand, modelling the role of diffusion sources can mine the latent topic of information. The diffusion sources can indicate the topic of the information [35]. In social network, as shown in Figure 1(c), most of the tweets by government officers are about politics; however, the actors always tweet some posts about travel and entertainment. In the meantime, users interested in the similar latent topic will have similar forward action which can help information cascade prediction. Similarly, in academic network, the scholars have their own research interests, and their work is usually cited by researchers who work in the similar research fields. In this paper, we are dedicated to mining the semantics of diffusion sources to help information cascade prediction, and Figure 1(a) shows the difference between our work and the previous work.

However, there are series of challenges to model the semantics of diffusion sources. Firstly, it is usually hard to collect the profiles of diffusion sources because of the privacy policy. How to model the diffusion sources without the explicit profiles is a problem. Then, the interaction between the users and diffusion sources is complicated. The influential diffusion sources have larger influence on users while the ordinary sources have smaller influence. Besides, different users behave differently when facing different diffusion sources. Therefore, it is a challenge to model the complex interaction from diffusion data. Finally, the distribution of diffusion sources is long-tailed. As shown in Figure 2, most of the information cascades come from a small part of diffusion sources. The imbalance distribution will lead to the bias of model; because of the sufficient cascade data from head sources, the latent semantics of head sources can be learnt better. In contrast, the tail sources perform significantly worse. For this reason, it is hard to learn the latent semantics of tail sources which is the majority in diffusion sources.

To address these challenges above, in this paper, we propose DSSF, a diffusion sources latent semantics-fusion framework. The framework consists of three parts: firstly, for modelling the heterogeneity of different diffusion sources, we introduce diffusion sources embedding for each user who acts as a diffusion source. Without explicit user profiles, the sources embedding learns the latent topic and diffusion pattern of the corresponding information cascades, which can facilitate information cascade prediction. Then, to learn the complicated interaction between users and diffusion sources, we propose a co-attention based fusion network to model how different diffusion sources affect users. Finally, to alleviate the data imbalance among the diffusion sources, we introduce an adversarial training framework to transfer the semantics knowledge from the well-trained head sources to tail sources.

In general, our contributions are three-fold as follows:

- To the best of our knowledge, we are the first to model the latent semantics of diffusion sources in the information cascade prediction problem.
- We introduce diffusion sources embedding and propose a co-attention based fusion gate to model the latent semantics of diffusion sources. We also study the effect of the diffusion sources distribution to our model and develop an adversarial training framework to alleviate the data imbalance problem. Our proposed framework can be widely adopted on existing diffusion prediction models such as RNN, LSTM, DeepDiffuse, and HiDAN. We will introduce the details in Section 4.
- We conduct experiments on two real-world datasets: Twitter and Weibo. The results show that modelling the diffusion sources can significantly improve the performance of various existing diffusion prediction models. The detailed experiment setting and results can be found in Sections 5 and 6.

## 2. Related Work

### 2.1. Information Diffusion Analysis

In 1927, Kermack [36] proposed the famous epidemic models to describe the trend of different groups. Epidemic models usually divide people into groups of S (Susceptible), I (Infected), and R (Recovered) and use a differential equation set to describe the change of number in each group. The rumour diffusion is similar to the spread of epidemic, and researchers carry out numerous studies of rumour diffusion and control with epidemic models. Epidemic models are group models which can only describe the trend of the whole group and ignore the network structure between users. Kempe [8] proposed influence diffusion models Independent Cascade (IC) and Linear Threshold (LT) and gave each node in the network status of active or inactive. At every moment, active users influence their neighbour users with a certain probability, and each user has only one chance to influence their neighbours. At last, the number of activated users in the network will converge. Furthermore, influence models are extended to continuous time and topic-aware [31]. Influence maximization is a typical study carried out based on the influence model [8, 37, 38].

### 2.2. Information Cascade Prediction

Information cascade prediction is an interesting and important topic in information diffusion analysis, which aims to capture and predict the tendency of information diffusion in the target network. The prediction can be divided into two aspects: cascade-level prediction and user-level prediction. Cascade-level prediction is to predict the overall trend of the diffusion in the target network, such as how many people will share the post [10, 18, 19, 39] or will this tweet be popular. User-level prediction focuses on the individual behaviour, such as who will be the next retweet user and when this user buys the goods. In the work, we focus on the user-level prediction and specifically on the next user prediction.

Traditional feature-based methods extract the features in information cascades, including time features, information items features, sequences features, and the social context features. However, the feature-based methods are time-consuming on feature engineering and have poor ability at fitting the data. Recently, with the fast development of deep learning techniques, researchers project diffusion cascade into a user sequence and formulate the user-level information cascade prediction as a sequence prediction problem. RNN and its variants (GRU [20] and LSTM [21]) are the typical deep learning architecture of sequence prediction. RNN-based models encode the historical user sequences into a fixed-length vector and predict the next active user through a fully connected network layer. RNN and its variants are simple but not good at modelling the long-term dependency and suffer from cross-dependence problem. Cross-dependency problem is caused by the tree structure in information diffusion and the user sequences. DeepDiffuse [12] introduces attention mechanism and sliding windows to help concentrate on the part most important to prediction. CYANRNN [27] uses a seq2seq model to predict the next active user step by step. Besides, self-attention models such as DAN [25] and HiDAN [26] are more efficient and perform better in capturing the cross dependence in diffusion sequences.

Besides, social relationship is the foundation communication channel between users. Users who are friends usually have common preferences and stronger pairwise social influence; thus, the social relationship between users is also important for information cascade prediction. Some models integrate the social context features such as the following relationship into deep sequences models: TopoLSTM [13] designs a dedicated RNN architecture for directed acyclic graph. SNIDSA [28] proposes a structural attention module to leverage the social relation, and FOREST [40] uses graph convolutional network [29] to aggregate the second-order neighbour features. DNRL [41] designs a jointly learning framework to learn user embedding from diffusion sequences and social network simultaneously. Besides, reference [42] focuses on the community structure in social network to help cascade prediction.

Previous deep learning-based information cascade prediction studies are committed to extracting the chronological features and cross-dependency. The heterogeneity of information items is not considered. It means that all the information cascade with the same preceding user sequences will have the same next user, which is unreasonable, especially when the preceding sequences are short. However, few of them pay attention to the effect of diffusion sources. Our work is to model the role of diffusion sources and propose an adversarial training strategy to focus on the tail information cascades.

## 3. Problem Formulation

Firstly, we give a formal definition of the basic concepts as follows.

### 3.1. Information Cascade

An information cascade is a user sequence ordered by user's infected time. Formally, given an user set, an information cascade can be represented as a user set ordered by the forward time *S*_*k*_={*u*_*k*_^0^, *u*_*k*_^1^,…, *u*_*k*_^|*S*_*k*_|−1^}, where |*S*_*k*_| is the length of cascade *S*_*k*_ and ∀*u*_*k*_^*t*^ ∈ *V*, 0 ≤ *t* ≤ *T*_*k*_.

### 3.2. Information Cascade Prediction

Given the information cascades training set *S*={*S*_1_, *S*_2_,…, *S*_*N*_}, a model *M*(*S*) is learnt to predict which user will be active at the next time, s.t. predict *u*_*t*_^|*S*_*t*_|^ of a test cascade instance *S*_*t*_={*u*_*t*_^0^, *u*_*t*_^1^,…, *u*_*t*_^|*S*_*t*_|−1^}. In this work, we focus on user activation prediction and take no account of the activation time.

Our goal can be divided into two parts. Firstly, we need to model the latent semantics hidden in the diffusion sources to support information cascade prediction. Secondly, we need to solve the difficulty caused by the long-tailed distribution of diffusion sources. Because of the data imbalance problem, the latent semantics of tail diffusion sources is difficult to learn directly from training data. Our objective is to transfer the semantics knowledge from the head sources to tail sources. We formally state our objectives as follows.

Given a training set *S*={*S*_1_, *S*_2_,…, *S*_*N*_}, for each information cascade *S*_*k*_={*d*_*k*_, *u*_*k*_^1^,…, *u*_*k*_^|*S*_*k*_|−1^}, the first user *u*_*k*_^0^ is the diffusion source and is denoted as *d*_*k*_. A model *M*(*d*, *S*) is learnt to predict which user will be active at the next time in a test cascade instance when the diffusion source is *d*.

Given the cascades from head diffusion sources *d*_*H*_ and tail sources *d*_*T*_, we also aim to strike the balance between the modelling ability of *d*_*H*_ and *d*_*T*_ by leveraging an adversarial training strategy.

## 4. Method

In this section, we will introduce a Diffusion Source Semantics-Fused (DSSF) cascade prediction framework. DSSF is composed of a diffusion source embedding layer, a co-attention-based fusion gate, and an adversarial training strategy, which can widely be adopted to different existing deep cascade prediction models. DSSF models the special role of diffusion sources with diffusion source embedding and fuses the semantics of ordinary user and diffusion sources by a co-attention fusion gate. Furthermore, to overcome the problem that the distribution of diffusion sources is imbalanced, we proposed an adversarial training strategy to transfer the knowledge learnt from head diffusion sources to tail diffusion sources.

### 4.1. Diffusion Sources Embedding

The diffusion sources act as a special role different from the ordinary users involved in information diffusion which can indicate abundant latent semantics including the potential activated user group and the latent topic of information. For modelling the heterogeneity of diffusion sources and incorporating the abundant latent semantics behind the sources, we introduce a diffusion sources embedding layer. For each diffusion source, a root user in social network or an author in academic network, we use a latent vector to represent its semantic feature and co-train with the user embedding. For jointly utilizing the semantics of users and diffusion sources, a direct method is to use the summation of the user embedding **u** and the diffusion source embedding **s** as the diffusion sources-fusion embedding.

(1) $$\begin{array}{c} {\tilde{u}}_{i}^{j}=u_{i}+s_{j}. \end{array}$$

We denote our model with this fusion method as DSSF_sum_.

### 4.2. Co-Attention-Based Fusion Gate

The direct summation operation does not consider the high-level relationship between users and diffusion sources. The diffusion behaviour of some users can be affected mainly by the diffusion sources but some users might be more affected by their predecessor users. Thus, we proposed a co-attention fusion gate to model how much each diffusion source affects users in forwarding decisions. The architecture of co-attention fusion gate is shown in Figure 3. Different from the summation fusion strategy, we design a co-attention layer which adopts bilinear attention mechanism [22] to calculate the attention scores between diffusion sources and users as follows:

(2) $$\begin{array}{c} a_{ij}=\frac{u_{i}W_{a}s_{j}{}^{T}}{\sum_{k=1}^{n}u_{i}W_{a}s_{k}{}^{T}}, \end{array}$$

where **W** ∈ *R*^*d*×*d*^ matrix and *a*_*ij*_ indicates how user *u*_*i*_ is influenced by diffusion source *d*_*j*_. After obtaining the attention score between user *u*_*i*_ and diffusion sources *d*_*j*_, we use a fusion gate to update the user embedding *u*_*i*_ under the diffusion source *d*_*j*_. Finally, we get the diffusion source semantics-fused user embedding as follows:

(3) $$\begin{array}{c} {\tilde{u}}_{i}^{j}=\left(1-a_{ij}\right)\cdot u_{i}+a_{ij}\cdot s_{j}. \end{array}$$

We update the user embedding in the deep diffusion prediction model to the diffusion source semantics-fusion embedding. We learn the latent semantics of diffusion sources by co-training the sources embedding with the base prediction model. It should be pointed out that our fusion method can be widely adopted to various deep diffusion prediction models which use embedding to represent each user.

We denote our model which adopts co-attention fusion gate as DSSF_att_.

### 4.3. Adversarial Training

Though the co-attention-based fusion gate can extract the latent semantics between users and diffusion sources, the long-tailed distribution causes the under-fit problem for tail diffusion sources. The co-attention function will be largely dominated by the head sources because the head sources have abundant training examples to learn the latent semantics. It will cause that the diffusion sources embedding and fusion gate only work for the head diffusion sources while for the tail data, the attention score in equation (2) will be approximate 0 and degenerate to the vanilla cascade prediction model.

While fortunately, there are some latent semantics which can be shared between head sources and tail source. For example, if the cascade sequences features from two diffusion sources are similar, the distance of these two sources should be close in embedding space. It means that we can transfer the knowledge from the head sources to the tail sources to alleviate the problem caused by data imbalance. Inspired by [43], for alleviating the problem caused by the long-tailed distribution of diffusion sources, we develop an adversarial training strategy to align the space of the diffusion sources-enhanced sequences encoding. Adversarial learning is firstly proposed to generate fake samples from random input as similar to the real images as possible [44]. Here, we adopt adversarial learning to transfer the latent semantics knowledge from the head to tail the cascades.

The architecture of adversarial training framework is shown in Figure 4. Besides the cascade prediction model, we introduce a discriminator to distinguish whether the cascade sequences encoding from head sources or tail sources. We denote the cascade encoder enhanced by our proposed fusion network as *E*(·;Θ_*e*_) and the prediction layer combined of a full-connected layer and a softmax function as *F*(·;Θ_*f*_). The discriminator is noted as *D*(·;Θ_*d*_). We want the discriminator to effectively distinguish where the cascade sequences are from, and we train the discriminator by minimizing the classification loss. In the meantime, the prediction model should generate the sequences encoding, which can fool the discriminator to misclassify and minimize the cascade prediction loss simultaneously. When the discriminator cannot differentiate the instance from head or tail, the latent space of the cascades sequences encoding is aligned.

We first divide the cascade sequences *S* into two categories according to the number of their diffusion sources and use 1 to indicate the head sources while 0 to indicate tail sources. The optimization object designed for adversarial training is composed of two parts: the cascade prediction loss and the discriminator loss. For the cascade prediction loss, we want to minimize the loss between the predicted results *F*(*E*(*x*;Θ_*e*_);Θ_*f*_) and real labels *y*. Each dimension of the predicted results *F*(*E*(*x*;Θ_*e*_);Θ_*f*_)_[*i*]_ indicates the probability of *u*_*i*_ being the next active user, and *y*_*i*_=1 indicates that *u*_*i*_ is the ground truth user. We use the cross-entropy loss same as the previous study [12, 13] as follows:

(4) $$\begin{array}{c} L_{\mathrm{prediction}}=E_{x∼P_{S}}-\log\sum_{i=1}^{N}y_{i}\cdot F{\left(E\left(x;\Theta_{e}\right);\Theta_{f}\right)}_{\left[i\right]}, \end{array}$$

where *N* is the number of the users.

For the discriminator loss, we first use the diffusion source semantics-fused cascade encoder layer to encode the sequence *x* into a vector *E*(*x*;Θ_*e*_). Our discriminator should distinguish the information cascade sequences from head sources *S*_*h*_ or tail sources *S*_*t*_. We use a binary cross-entropy loss as follows:

(5) $$\begin{array}{c} L_{\mathrm{discriminator}}=E_{x∼P_{S_{h}}}-\log D\left(E\left(x;\Theta_{e}\right);\Theta_{d}\right)+E_{x∼P_{\mathrm{St}}}-\log D\left(E\left(x;\Theta_{e}\right);\Theta_{d}\right). \end{array}$$

For aligning the vector space of information cascade and minimize the prediction loss simultaneously, we introduce a gradient inverse layer before the discriminator [43] and we optimize the model with a minimax object as follows:

(6) $$\begin{array}{c} \underset{\Theta_{e},\Theta_{f}}{\min}\underset{\Theta_{d}}{\max}L_{\mathrm{prediction}}-\lambda L_{\mathrm{discriminator}}, \end{array}$$

where *λ* is a hyperparameter to balance the cascade prediction and the knowledge transfer. Specifically, the adversarial training process is summarized in Algorithm 1. The discriminator is trained every *k*_*d*_ epochs to distinguish whether the cascade sequences from head or tail sources (line 7-8). Meanwhile, the diffusion source semantics-enhanced encoder is trained to maximize the classification loss of the discriminator (line 10) and minimize the cascade prediction loss simultaneously (line 11).

Compared with setting a fixed value of *λ* [43], we believe that an adaptive strategy with a warm-up strategy can have better effect. At the early stage of training, *λ* should be small to make sure the model learns from head data sufficiently. As the training goes on, *λ* should be larger and make our training focus on the knowledge transferring. Thus, we propose an adaptive exponential growth strategy with a warm-up as follows.

(7) $$\begin{array}{c} \lambda =\left\{\begin{array}{cc} \mathrm{0,} & k<K_{0},\\ 1-e^{\left(K-k\right)}, & k\geq K_{0}, \end{array}\right) \end{array}$$

where *K* is the total number of epoch and *K*_0_ is the warm-up number of the epoch.

## 5. Experiments

In this section, we will introduce the datasets, baseline methods we will compare with, the metrics we adopt, and the detailed experiment setting such as data preprocessing and the hyperparameters.

### 5.1. Dataset

#### 5.1.1. Twitter

Twitter [45] dataset records the URLs sharing among users in Twitter, a microblogging platform on which millions of Twitter users can share the short messages with each other [39]. The dataset is sampled from the URLs sharing from Mar 24 to Apr 25 in 2012. Each URL is an information, and the URL sharing among users forms an information cascade. We treat the first user who created the URL as diffusion source. The Twitter dataset includes 5942 users, and the average length of the cascades is 17.0422.

#### 5.1.2. Weibo

Weibo [46] dataset records the retweet behaviours in a popular microblogging platform: Sina Weibo. The retweet behaviours among users in Sina Weibo form the information cascades, and the users who post the content are the diffusion sources. The dataset contains 8183 users and 39029 cascades with an average cascade length of 21.9078.

The statistics data of two social network datasets are shown in Table 1.

### 5.2. Baselines

#### 5.2.1. RNN

RNN is a typical network architecture in sequence modelling, which can encode the historical information into a fixed vector with the following equations:

(8) $$\begin{array}{c} h_{t}=\tanh\left(W\cdot \left[h_{t-1},x_{t}\right]\right)+b_{h},\\ o_{t}=V\cdot h_{t}+b_{o}. \end{array}$$

#### 5.2.2. LSTM

LSTM [21] is a variant of RNN, which is widely used in sequence modelling. LSTM adopts gate mechanism to solve the gradient vanishing and gradient exploding problems which appear in training long sequences. LSTM is composed of input gate, forget gate, and output gate. Each gate can choose what information should be preserved. The inference equation of LSTM cell is as follows:

(9) $$\begin{array}{c} f_{t}\mathrm{=\sigma}\left(W_{f}\cdot \left[h_{t-1},x_{t}\right]+b_{f}\right),\\ i_{t}\mathrm{=\sigma}\left(W_{i}\cdot \left[h_{t-1},x_{t}\right]+b_{i}\right),\\ {\tilde{C}}_{t}=\tanh\left(W_{C}\cdot \left[h_{t-1},x_{t}\right]+b_{C}\right),\\ C_{t}={\tilde{C}}_{t}⊙i_{t}+f_{t}⊙C_{t-1},\\ o_{t}\mathrm{=\sigma}\left(W_{o}\cdot \left[h_{t-1},x_{t}\right]+b_{o}\right),\\ h_{t}=o_{t}⊙\tanh\left(C_{t}\right). \end{array}$$

#### 5.2.3. DeepDiffuse

DeepDiffuse [12] predicts not only which node will be infected but also when the user will be infected. In this work, we only focus on the user prediction part in DeepDiffuse. Comparing with vanilla LSTM, DeepDiffuse brings attention mechanism [22] and sliding windows for a more flexible model.

#### 5.2.4. HiDAN

HiDAN [26] is a nonsequence diffusion prediction model which replaces the recurrent layer with the hierarchical self-attention [24], which can capture historical cross-dependencies and time-decay effects between users. HiDAN is much faster than RNN-based models because the attention computation is easier to parallelize.

### 5.3. Evaluation Metrics and Setting

Because the number of potential active users is large, the diffusion prediction is usually viewed as an information retrieval problem. We need to query the rank of the next active user given the probability of all the users. The model is better if the predicted node has a higher rank. We adopt two widely used evaluation metrics in diffusion prediction:

- Hit@k is the rate of top *k* ranked nodes containing the next active node. The larger Hit@k indicates the better predictive ability of the candidate forward users groups.
- MRR is the Mean Average Precision which is commonly used in information retrieval. Above the hitting rate in top *k*, MRR considers the rank of the next node in ranked nodes simultaneously. The larger MRR indicates the predicted nodes have higher rankings.

For the data processing, we randomly divide the dataset into training, valid, and testing dataset according to the proportion of 80%, 10%, and 10%. We truncate the cascade sequence at the max length of 100. We implement all our models with deep learning framework Pytorch [47]. For HiDAN and DeepDiffuse, we use the time-free version, which takes no consideration of time. For the training detail, the hidden size of all the models is set to 64 same as the setting in HiDAN. The learning rate of the diffusion prediction model and domain classification model is 0.001, and we use Adam [48] as the optimizer.

## 6. Results

In this section, we will show that our proposed model significantly performs better than the competitive methods. We firstly present the overall results on information cascade prediction. Then, we conduct series of ablation studies to show the effectiveness of our model. Finally, we summarize our findings concluded from our results.

### 6.1. Evaluation

We conduct experiments on two social network datasets Twitter and Weibo and use RNN, LSTM, DeepDiffuse, and HiDAN as the baseline models. We adopt DSSF on above four baseline models, respectively, and each of the improved models is denoted as RNN + DSSF, LSTM + DSSF, DeepDiffuse + DSSF, and HiDAN + DSSF. The results are shown in Table 2, and for each model, the first line records the results of the original model, the second line records the results of the improved model, and the third line records the relative improvement of the improved model.

From the evaluation results, we find that our method can perform better on both MRR and Hit@k, respectively, than all the compared methods. For the Twitter dataset, the improvement of DSSF on MRR ranges from 3.16% to 8.04% and the improvement of Hit@K is more obvious which is from 4.01% to 23.39%. For the Weibo dataset, the improvement of DSSF on MRR is more significant than Twitter, which is from 7.38% to 21.01%. However, the improvement on Hit@k is not that obvious, which is from 6.38% to 15.75%.

From the results, we can conclude two aspects. Firstly, for both datasets, the improvement is significant on different baseline models. This result shows that our proposed method modelling the diffusion sources can indeed help the information cascade prediction. Secondly, the improvement to Twitter and Weibo is different, which shows that the effect of diffusion sources is different in different scenes. In the Twitter dataset, the gain on Hit@k is more significant. It means that modelling the diffusion sources helps more in potential users group prediction in the Twitter dataset. However, in the Weibo dataset, the promotion on the MRR is greater than Hit@k, which indicates that diffusion sources help more in the rank of predicted users.

### 6.2. Ablation Study

Compared with the baseline models, DSSF learns the latent semantics with a co-attention fusion gate and alleviates the data imbalance problem with an adversarial training framework. Here, we do further analysis. Does the diffusion sources embedding work? How does the fusion gate impact the latent semantics learning? Whether the adversarial training help in knowledge transfer? To answer these questions, we conduct ablation studies from two aspects: (a) on the one hand, we replace the diffusion source embedding **S** with user embedding **U** to evaluate whether the diffusion sources embedding can model the special role of root users. We note the model as DSSF_user_. One the other hand, DSSF_sum_ we introduce in Section 4 sums the user embedding and diffusion source embedding, which introduces the diffusion sources information but does not consider the high-level semantics information. We compare the DSSF_att_ version with DSSF_sum_ and show that how well our fusion gate learns the semantics. In this part, we use LSTM as the base models. (b) We take Twitter dataset as an example to compare the model without adversarial training and give a more detailed analysis according to the distribution of diffusion sources.

From the results shown in Figure 5, we can see that DSSF_user_ can significantly improve the performance on the hit@50 and hits@100 in Twitter datasets comparing with the base models, which means that the modelling diffusion sources can effectively handle the potential forwarding user group in information diffusion. And in the meantime, the DSSF_sum_ models the special role of diffusion sources without consideration of the latent interaction with users which has great improvement on MRR and hits@10 on both datasets. The results of DSSF_sum_ mean that modelling the special role of diffusion sources significantly captures the cascade prediction. Furthermore, the DSSF_att_ performs better than both DSSF_user_ and DSSF_sum_ which shows that modelling the latent interaction between users and diffusion sources can help describe more details in information diffusion.

The results in Figure 6 show the prediction performance on the cascades from tail diffusion sources. We conduct experiments on Twitter dataset with four base methods. The DSSF model without “NA” means training with adversarial strategy, while models with “NA” mean training with only the prediction loss. From the results, we can see both the MRR and Hit@k have obvious improvement on the tail cascades, which shows that the adversarial training strategy can effectively improve the prediction on tail cascades. It means that the semantics knowledge transfer from the head to tail cascades with the adversarial training framework.

### 6.3. Discussion

The results of our experiments above show that diffusion sources act as a special role in information diffusion which is different from ordinary users, and the abundant information behind source users can be used to help cascade prediction. Specifically, our findings can be divided into three parts as follows:

1. We find that abundant latent semantics hidden behind the diffusion sources can help information cascade prediction, which is ignored by most existing methods. The experiment results in Table 2 show that our proposed framework which aims to model latent semantics of diffusion sources can significantly improve the prediction performance comparing with the existing models treating diffusion sources as ordinary users.
2. Further, we find that the model with a co-attention-based fusion gate performs better than the summation fusion model from the results shown in Figure 5. The results indicate that the interaction between users and diffusion sources is different from user to user,
3. Finally, from the results in Figure 6, we find that the adversarial training framework can effectively improve the performances of cascades from tail diffusion sources. The results show that the semantics knowledge in different diffusion sources is transferable, and we can solve the difficulty caused by data imbalance with adversarial learning framework.

## 7. Conclusions

In this paper, we study the special role of diffusion sources in information diffusion and propose DSSF, a diffusion source semantics-fused cascade prediction framework to learn the latent semantics between users and diffusion sources. Our framework consists of two parts. The co-attention-based fusion gate is to learn the special role of diffusion sources as well as the latent interaction between users and sources. However, the long-tailed distribution of diffusion sources will cause little improvement on the tail cascades. The second part of our framework is for this problem. We develop an adversarial training strategy to transfer the semantics knowledge from the head cascades to the tail. The experiment results show that our framework can effectively learn the latent semantics for both head and tail cascades.

In the future, we will further extend our framework to the diffusion prediction model with consideration of the time-decay effect, social context, and information content. We will also explore the high-order semantics between users and diffusion sources. For example, multiple users who have forwarded information from the same diffusion sources will have similar actions.

## Figures and Tables

**Figure 1:** Modelling the diffusion sources. (a) Previous work focuses on modelling the cascade sequences but ignores the diffusion sources. (b) Diffusion source is an important factor of forwarding decision. (c) Tweets from one diffusion source have similar topic.

**Figure 2:** Long-tailed distribution of diffusion sources.

**Figure 3:** The architecture of the co-attention fusion gate. The fusion gate is composed of embedding layer, co-attention layer, and fusion layer. (1) The embedding layer transforms diffusion sources and users into two different embedding spaces. (2) The co-attention layer extracts the interaction between users and diffusion sources with bilinear attention mechanism. (3) The fusion layer aggregates the semantics of users and diffusion sources together in support of the further cascade prediction.

**Figure 4:** The diagram of adversarial training framework. Firstly, the cascade sequences are divided into two categories according to the cascade sequences number of their diffusion sources. Secondly, the cascade sequences are encoded with the encoder-based cascade prediction model. Finally, the model is trained in an adversarial paradigm which minimizes the cascade prediction loss and meanwhile maximizes the discriminator loss.

**Figure 5:** Ablation study on Twitter and Weibo datasets.

**Figure 6:** Performance on cascades from head and tail sources.

**Algorithm 1:** Adversarial training framework in DSSF.

**Table 1:** Statistics of evaluation datasets.

Dataset	# Users	# Diffusion sources	# Cascades	Average cascade size
Twitter	5942	204	569	17.0422
Weibo	8183	6541	39029	21.9078

**Table 2:** Evaluation results on Twitter and Weibo datasets.

Method/gain	Twitter				Weibo			
	MRR	Hit@10	Hit@50	Hit@100	MRR	Hit@10	Hit@50	Hit@100
RNN	21.37	23.82	25.93	27.19	1.76	2.82	8.09	13.17
**RNN** + **DSSF**	**23.03**	**26.77**	**31.81**	**33.55**	**1.89**	**3.00**	**8.73**	**14.05**
Gain	**8.04**	**12.38**	**22.68**	**23.39**	**7.38**	**6.38**	**7.91**	**6.68**
LSTM	21.82	26.17	28.45	29.41	1.38	2.74	8.89	14.59
**LSTM** + **DSSF**	**23.51**	**28.59**	**33.25**	**35.11**	**1.67**	**3.15**	**9.73**	**15.75**
Gain	**7.75**	**9.25**	**16.87**	**19.38**	**21.01**	**14.96**	**9.45**	**7.95**
DeepDiffuse	18.34	25.93	28.63	29.89	1.61	3.06	9.78	15.84
**DeepDiffuse** + **DSSF**	**18.92**	**26.97**	**32.41**	**34.45**	**1.89**	**3.37**	**10.21**	**17.27**
Gain	**3.16**	**4.01**	**13.20**	**15.25**	**17.39**	**10.13**	**4.39**	**9.02**
HiDAN	22.34	25.87	28.51	29.41	1.90	3.54	10.03	15.86
**HiDAN** + **DSSF**	**23.11**	**27.67**	**32.11**	**34.84**	**2.11**	**3.83**	**11.31**	**17.12**
Gain	**3.46**	**6.95**	**12.62**	**18.46**	**11.05**	**8.19**	**12.76**	**7.94**

## Data Availability

The data used to support the findings of this study are included within the article.
